The article "Clinical Study of Intravitreal Injection of Anti-VEGF Drugs Combined with Triamcinolone Acetonide in the Treatment of Coats Disease" was retracted in 2023. Reasons: unreliable results or conclusions; lack of ethics approval or compliance; concerns about the data; concerns about the peer review.

# Clinical Study of Intravitreal Injection of Anti-VEGF Drugs Combined with Triamcinolone Acetonide in the Treatment of Coats Disease

**DOI:** 10.1155/2022/9911549

**Published:** 2022-06-17

**Authors:** ShaoFeng Wu, Jing Fang, Fang Yu, Fang Han, Jun Xiao

**Affiliations:** ^1^Department of Ophthalmology, Huangmei People's Hospital, 137 Wuzu Dadao, Huangmei Town, Huangmei County, Huanggang City, Hubei Province 435500, China; ^2^Anesthesiology Department, Caidian District People's Hospital of Wuhan, No. 111 Chenggong Avenue, Caidian District, Wuhan City, Hubei Province 430100, China; ^3^Shenzhen Hospital, University of Chinese Academy of Sciences (Guangming) (Ophthalmology), 39 Huaxia Road, Guangming Street, Guangming District, Shenzhen City, Guangdong Province 518107, China; ^4^Xiangyang Integrated Traditional Chinese and Western Medicine Hospital/Ophthalmology, No. 16, Dongfeng Automobile Avenue, High Tech Zone, Xiangyang City, Hubei Province 411000, China; ^5^Eastern Hubei Medical Group City Maternal and Child Health Hospital Ophthalmology, 9 Guilin South Road, Xialu District, Huangshi City, Hubei Province 435000, China

## Abstract

**Objective:**

To investigate the clinical study of intravitreal injection of anti-VEGF drugs combined with intravitreal injection of tretinoin for the treatment of Coats disease.

**Methods:**

The medical records of 90 patients (120 eyes) with Coats disease admitted to our hospital from April 2010 to June 2021 were selected as retrospective study subjects and divided into control and treatment groups according to the numerical table method. There were 45 cases and 60 eyes in each group. Among them, intravitreal tretinoin drug was injected into the control group, and anti-VEGF drug was injected into the vitreous sclera of the treatment group on the basis of the control group.

**Results:**

Before treatment, the differences in visual acuity changes between the two groups were not statistically significant (*P* > 0.05). After treatment, the light perception, manipulation, and indexes of both groups were significantly improved, and the treatment group was significantly better than the control group. This difference was statistically significant (*P* < 0.05) for statistical study comparison. The effective rate of 95.56% in the treatment group was significantly higher than that of 86.67% in the control group, and the complication rate was significantly lower than that of the control group, with statistically significant differences (*P* < 0.05).

**Conclusion:**

Intravitreal injection of anti-VEGF drugs combined with tretinoin injection can significantly improve the clinical efficacy of patients with Coats disease and improve visual acuity and central retinal thickness, which has certain reference value for the clinical treatment of Coats disease.

## 1. Introduction

Coats disease is the outer layer of exudative retinopathy, which is mostly manifested as secondary telangiectasia, which often leads to monocular invasion [1]. The course of the disease is slow and has progressive characteristics. Some patients may have concurrent symptoms such as cataracts, glaucoma, and low intraocular pressure, which have adverse effects on the normal function of the eye [2]. The pathogenesis is still unclear. Some scholars have performed tests on patients with antibodies against multiple pathogens, blood routines, serum angiotensin-converting enzymes, and antinuclear antibodies. No abnormalities were found. Therefore, they think it may be a kind of myopia, caused by degenerative diseases [3]. However, the patient shows an inflammatory response, and it is difficult to explain the clinical manifestations of the patient with the viewpoint of degeneration [4]. Coats disease is mostly manifested as secondary telangiectasias, which often leads to monocular invasion. The course of the disease is slow and progressive. Some patients may be complicated by symptoms such as cataract, glaucoma, and low intraocular pressure and have adverse reactions to the normal function of the eye [5]. At present, the clinical treatment of Coats disease has not yet reached a consensus. Intravitreal injection of drugs is considered to be one of the first choices for the treatment of Coats disease, but there is still some controversy in the choice of drugs [6]. Based on this, in order to explore the clinical efficacy of intravitreal injection of anti-VEGF drugs combined with intravitreal injection of triamcinolone acetonide in patients with Coats disease, our hospital has conducted certain explorations. The current research results are reported as follows. This study investigated the clinical efficacy of intravitreal trimethoprim in patients with Gauss' disease and showed improvements in visual acuity and central retinal thickness. Trimethoprim can inhibit the proliferation of capillary endothelial cells induced by fibroblast growth factor (bFGF), thereby inhibiting the formation of neovascular membranes. It has a long half-life in the eye, and some studies have shown that intravitreal triamcinolone acetonide maintains certain concentrations in the eye for four months after intravitreal injection. However, this is still not an option for economically disadvantaged patients. As the research on antivascular endothelial growth factor drugs continues to deepen, its unique benefits for choroidal neovascular disease are becoming more and more obvious. Vascular endothelial growth factor (VEGF) activates its receptors, causes angiogenesis, and affects vascular permeability through a series of responses.

## 2. Materials and Methods

### 2.1. General Information

We selected 90 patients (120 eyes) with Coats disease who were treated in our hospital from April 2010 to June 2021 as the subjects of this prospective study and were divided into a control group and a treatment group with 45 cases each (60 eyes). Diagnosis of Coats disease: the patient has symptoms such as neck stiffness, dizziness, and limb weakness; the patient's cervical spine itself has tenderness; the patient's activity will aggravate the condition. Differences in general clinical data such as gender, age, and body mass index of the two groups of patients have no effect on this study (see Table 1 for details).

### 2.2. Standards for Inclusion and Exclusion

Inclusion criteria are as follows: (a) all patients in this study met the “Polypoidal choroidal vasculopathy: evidence-based guidelines for clinical diagnosis and treatment” [7] Western medical diagnostic criteria for Coats disease. (2) The edge of the optic disc (abnormal new blood vessels exist in the area around the optic papilla) involves the central area of the macula. (3) The patient's visual acuity is equal to 20/320 to 20/25 of the Snellen visual acuity chart. Exclusion criteria are as follows: (1) patients have hypertension (>140/90 mmHg), high intraocular pressure (IOP = 24 mmHg), and hypersensitivity and have a history of stroke or myocardial infarction within 3 months. (2) Patients used other study drugs within 30 days and use systemic glucocorticoids or anti-VEGF drugs within 6 months. (3) The patient has any active eye infection, active intraocular inflammation, iris neovascularization or neovascular glaucoma, history of uveitis, and vitreous macular traction syndrome; cannot obtain sufficient quality fundus photographs or fluorescein angiography for analysis; and uses any hormones and antiangiogenic drugs (including any glucocorticoids and anti-VEGF drugs) within 3 months.

### 2.3. Treatment Methods

The control group was treated with intravitreal injection of triamcinolone acetonide. The method of operation is as follows: disinfection of drapes, eyelid opener, elcaine eye drops for superficial anesthesia, and 27# needle disposable. A 1.0 mL empty needle withdraws a 0.1 mL dose of triamcinolone acetonide suspension (drug concentration of 40.0 mg/mL), and the needle was inserted 4.0 mm behind the limbus of the subtemporal cornea, and the drug is injected into the vitreous cavity. After the injection, the patient's intraocular pressure is checked. If the intraocular pressure is higher than the normal level, the anterior chamber puncture is performed simultaneously to reduce the intraocular pressure. Erythromycin was evenly applied to the conjunctival sac, and antibiotic eye drops were used for eye drops at the second hour after the operation, with a frequency of 3 times per day. In the treatment group, on the basis of the control group, the anti-VEGF drug was injected into the vitreous and sclera. The operation method is exactly the same as that of the control group. After superficial anesthesia, a 1.0 mL empty needle with a 27# needle was used to withdraw 0.05 mL of anti-VEGF injection, and the needle was inserted 4.0 mm behind the infratemporal corneal limbus, and the drug was injected into the vitreous cavity.

### 2.4. Observation Indicators

(1) The ocular surface disease index (OSDI) was measured before and after treatment to total 100 points. The lower the score, the lighter the patient's symptoms. (2) Efficacy evaluation: that is effective: the patient's symptoms and signs are completely relieved or disappeared. Improvement: partial relief of symptoms and signs. Ineffective: no improvement in symptoms and signs. Effective rate = (effective + improvement) × total number of cases.

### 2.5. Statistical Methods

Use Epidata to enter all the data, and then, use SPSS 25.0 to statistically process the data. The data needs to be entered into the computer database by a second person to ensure the completeness and accuracy of the data. The independent sample *t*-test was used to express the measurement data in terms of mean ± standard deviation ($\bar{x}\pm S$), and the count data in percentage (%) was used to use the *χ*^2^ test. Statistical *P* < 0.05 indicated significant difference.

## 3. Results

### 3.1. Comparison of General Information

The comparison of general data such as gender, average age, course of disease, log MAR BCVA, and intraocular pressure between the two groups of patients showed no significant statistical difference after *t*-test and chi-square test (*P* > 0.05) (see Table 1).

### 3.2. Comparison of Vision Changes

Before treatment, the visual acuity changes of the two groups were not statistically significant (*P* > 0.05). After treatment, the light perception, manual, and index of the two groups were significantly improved, and the treatment group was significantly better than the control group. Statistical comparison: this difference is significant (*P* < 0.05) (see Table 2).

### 3.3. Comparison of Central Retinal Thickness and Self-Perceived Symptoms

Before treatment, the comparison of the central retinal thickness and conscious symptoms of the two groups of patients was not statistically significant (*P* > 0.05). After treatment, the central retinal thickness and OSDI of the two groups were significantly improved, and the treatment group was significantly better than the control group. This difference is statistically significant (*P* < 0.05) (see Table 3).

### 3.4. Analysis of Clinical Efficacy

The clinical efficacy analysis after treatment showed that the effective rate of 95.56% of the patients in the treatment group was significantly higher than that of the control group, 86.67%, while the complication rate was significantly lower than that of the control group. The difference was statistically significant (*P* < 0.05) (see Table 4).

## 4. Discussion

Patients with Coats disease may develop a range of complicating symptoms as their condition progresses, and some severely ill patients may eventually lose their vision [8]. Therefore, it is important to take active measures in clinical treatment to control the occurrence of retinal detachment and promote the improvement of patients' vision. The clinical value of tretinoin intravitreal injection in the treatment of Coats' disease has now been confirmed by some reports [9]. In previous studies, it was concluded that tretinoin relieved inflammatory symptoms in the eye, relieved capillary dilation, and had a good limiting effect on fibrin exudation, but it has also been shown that treatment with tretinoin intravitreal injection alone was difficult to stop the progression of the disease, and approximately 78% of patients with stage 4 Coats disease eventually required removal of the eye after conventional treatment, with serious irreversible consequences [10]. Intravitreal injection therapy with anti-VEGF drugs has a positive effect on improving vision in patients with Coats disease [11]. The analysis concluded that patients with Coats disease tend to have a high expression of VEGF in their eyes, and anti-VEGF drug treatment can effectively reduce the level of VEGF in patients' eyes, promote the regression of iris neovascularization, accelerate the absorption of subretinal fluid, and reduce the difficulty of surgery, thus avoiding the adverse outcome of Coats disease patients who eventually have their eyes removed due to the progression of the disease [12]. Trimethoprim is a non-water-soluble, long-acting glucocorticoid with strong anti-inflammatory effects [13]. Both domestic and international studies have now demonstrated that vitreous cavity injection of tretinoin is a safe and effective treatment for all causes of uveitis and aids vitrectomy to improve the success rate of surgery [14].

This study investigated the clinical efficacy of intravitreal trimethoprim in patients with Gauss' disease and showed improvements in visual acuity and central retinal thickness [15]. Trimethoprim counteracts fibroblast growth factor- (bFGF-) induced proliferation of capillary endothelial cells, thereby inhibiting the formation of neovascular membranes [16]. It has a long half-life in the eye, and some studies have shown that intravitreal tretinoin maintains a certain concentration in the eye after four months of intravitreal injection [17]. However, it is still not an option for patients with poorer economic conditions. As research on antivascular endothelial growth factor drugs continues, their unique benefits for choroidal neovascular disease are becoming increasingly apparent [18]. Vascular endothelial growth factor (VEGF) activates its receptors, causing vascular neovascularization and affecting vascular permeability through a series of responses [19, 20].

To sum up, conventional scleral withholding and external pressure-assisted vitreous injection of anti-VEGF drugs combined with intravitreal triamcinolone acetonide drug therapy can significantly improve the clinical efficacy of patients with Gaussian disease and improve visual acuity and central retinal thickness and the clinical treatment of Gaussian disease. There is a certain reference value.

## Figures and Tables

**Table 1:** Comparison of general information between the two groups [*n*, ($\bar{x}\pm s$)].

Group	Gender (men and women)	Average age (age)	Course of disease (year)	Log MAR BCVA	Intraocular pressure (mmHg)
Control group (45)	23/22	16.63 ± 3.32	1.31 ± 0.67	1.52 ± 0.25	9.75 ± 1.22
Therapy group (45)	24/21	15.62 ± 4.31	1.33 ± 0.25	1.54 ± 0.34	9.35 ± 2.57
*χ* ^2^/*t*	0.045	0.006	-0.188	-0.318	0.943
*P*	0.833	0.995	0.852	0.751	0.348

**Table 2:** Comparison of visual acuity changes between the two groups ($\bar{x}\pm s$).

Group	Light-sensitive		Manual		Index		>0.05		0.01~0.05	
	Before therapy	After treatment	Before therapy	After treatment	Before therapy	After treatment	Before therapy	After treatment	Before therapy	After treatment
Control group (45)	11	9	16	13	11	15	7	8	5	5
Therapy group (45)	10	6	17	8	11	18	7	10	5	8

Note: the comparison between groups before treatment is *P* > 0.05, and the comparison between groups after treatment is *P* < 0.05.

**Table 3:** Comparison of central retinal thickness and self-perceived symptoms between the two groups ($\bar{x}\pm s$).

Group	Central retinal thickness		OSDI	
	Before therapy	After treatment	Before therapy	After treatment
Control group (45)	289.74 ± 10.30	239.97 ± 15.39	18.24 ± 0.22	16.91 ± 3.07
Therapy group (45)	285.75 ± 14.33	261.83 ± 12.19	18.25 ± 0.23	12.77 ± 3.10
*t*	1.517	-7.469	-0.211	6.365
*P*	0.133	0.000	0.834	0.000

**Table 4:** Clinical efficacy of two groups of patients [*n* (%)].

Group	Efficient	Get better	Invalid	Efficient (%)
Control group (45)	19 (42.22)	20 (44.44)	8 (17.78)	39 (86.67)
Therapy group (45)	22 (48.89)	21 (46.67)	2 (4.44)	43 (95.56)
*χ* ^2^				4.050
*P*				0.044

## Data Availability

The raw data supporting the conclusions of this article will be made available by the authors, without undue reservation.
